The article "Construction of the Public Management Performance Assessment Algorithm Using Fuzzy Clustering" was retracted in 2023. Reasons: signs of a paper mill; suspected computer-generated content; unreliable results or conclusions; concerns about the data.

# Construction of the Public Management Performance Assessment Algorithm Using Fuzzy Clustering

**DOI:** 10.1155/2022/1272099

**Published:** 2022-08-02

**Authors:** Rong Zhang

**Affiliations:** School of Marxism, Hubei Polytechnic University, Huangshi 435003, China

## Abstract

This paper analyzes the limitations of the current public management performance evaluation system, puts forward a public management performance evaluation model based on fuzzy clustering, and expounds on the theoretical framework and principle of this method. In addition, this paper introduces the concept and method of public management performance evaluation into the evaluation content system of government under the rule of law and realizes the combination of government under the rule of law theory and public management performance evaluation methodology. At the same time, through the analysis of the organizational system, technical system, institutional mechanism, result orientation, public satisfaction, and related index content, a public management performance evaluation index system is designed. Through macro and micro, qualitative and quantitative analysis and evaluation, the performance evaluation index system is improved, which provides an objective basis for forecasting and decision-making, control, and adjustment. The research shows that the highest accuracy of this clustering method can reach about 96%, and its accuracy is about 10% higher than that of the ID3 algorithm. It is expected that this research can make some contributions to the research of the public management performance evaluation index system. At the same time, it highlights the importance of research on performance evaluation of government ruled by law.

## 1. Introduction

Where there is an organization, there is management and evaluation. “Promoting construction by evaluation” conforms to the incentive principle of management. It is a new attempt to apply the concept of performance evaluation to public management evaluation, a booster for the construction of a government ruled by law, and it has been recognized by more and more people [1]. The performance of public administration departments determines the overall level of national public administration, and the performance evaluation of public administration departments is an important problem of national public administration, which is of great significance to the political development of different countries. The effectiveness of public management and administrative execution of public functional departments, that is, how to objectively and comprehensively assess and evaluate the performance of public management and administrative execution and form a systematic performance management system of public functional departments, is one of the most discussed issues in the theoretical circle of public management in recent years [2]. Concept to action, local to global, public management is a complex system process. To improve public management, it is necessary to evaluate it. A question that warrants careful consideration by researchers is how to establish a set of scientific, reasonable, systematic, dynamic, practical, and operable public management evaluation systems based on the results of the available research and the actual situation [3]. An example of quantitative data is an index, which is a collection of statistical data. It is employed to describe the social condition index, carry out social planning and analysis, and assess both the present and the future. Establishing a public management performance evaluation index system that is characterized by legal standards, participation of the entire population, sound institutions, and scientific evaluation is of utmost importance, as is strengthening the cost accounting and performance evaluation of public management.

The operation mechanism of public management as a complex, enormous system has not been thoroughly and methodically clarified in prior research, and it is, therefore, unable to fully and dynamically reflect the current situation and trajectory of the object. As a result, there are inevitably some issues with the operability of evaluation, the design of the index system, the selection of evaluation targets, and the orientation of the evaluation object [4]. In addition, the complexity and uncertainty of public management make management extremely complex. The index system, which serves as the foundational component of public management performance evaluation, is a crucial requirement for its successful development [5]. The development of a rational and scientific index system to assess the efficacy of public management is a common and urgent need shared by the government, social organizations, and the general public. The indicators to be evaluated in the public management performance evaluation system cover a broad spectrum. The calculation of evaluation results is very difficult due to the completely different evaluation index weights, evaluation requirements, information sources for the evaluation data, calculation processes for the data, and quantitative indicators for the data. The fuzzy clustering method [6, 7] can help mitigate this issue to some extent. In addition, the current performance evaluation system lacks a strong theoretical foundation for the weight proportion distribution of each evaluation index. In this paper, a fuzzy cluster analysis-based performance evaluation model [8] for public management is proposed, along with an evaluation index framework. This makes it possible to analyze and evaluate public management objectively as a whole, and it gives managers a solid foundation on how to conduct public management in a rational and scientific manner. The innovation of this paper is as follows:

1. Taking the government under the rule of law as the research object, this paper expounds on the background and significance of the government under the rule of law, defines the connotation of the government under the rule of law, and analyzes in detail the evaluation index system and ideas of the government under the rule of law constructed by governments at all levels through material collection. Then, the concept and method of public management performance evaluation are introduced into the evaluation content system of government under the rule of law, and the combination of government under the rule of law theory and public management performance evaluation methodology is realized to derive a new concept category.
2. In this paper, the AHP (analytic hierarchy process) is improved, and the substitution indexes of single importance evaluation are compared pairwise so as to innovate the technical path of constructing the index system. At the same time, through the analysis of the organizational system, the technical system, the institutional mechanism, result orientation, public satisfaction, and the research of related indicators, an evaluation index system of first-level indicators and second-level indicators is finally designed. In addition, according to the empirical results, the index system is compared and tested by multiple schemes to enhance the scientificity and persuasiveness of the index system.

The performance evaluation model of public management based on fuzzy clustering is the main topic of this paper. The paper is organized as follows: The introductory part is the first section. This section provides information on the specific research subject, research context, and research significance. In addition, it introduces the paper's innovative research methodology and section structure. A related work is the second one. This section presents the research work and methods used in this paper, as well as the current state of the research on the research topic. The third section provides a brief overview of the pertinent theoretical underpinnings and proposes a fuzzy clustering-based performance evaluation model for public management. The experimental analysis the fourth section. The summary and prospect is the fifth one. The findings of this paper's research are compiled in this section. Finally, this paper's flaws are discussed, along with the direction future research should take.

## 2. Related Work

The main body of public management performance evaluation is the people, and the people are the judges of the evaluation results. Performance evaluation is an important way to evaluate the work behavior of different departments by scientific methods. At present, there are many research studies conducted on performance evaluation.

Gross et al. constructed using objective index evaluation, expert evaluation, and public satisfaction measurement in one of the rule of law government performance evaluation index systems. These systems are based on the logical starting point of target evaluation, based on the result orientation and public satisfaction orientation, as a special case of AHP, using the expert consultation and survey method [9]. After determining the index system of the school teacher performance evaluation system, Lee studied the general calculation method and safety and fairness measures and gave the calculation model of each index and the calculation model and algorithm implementation of the final evaluation score of teachers. A scientific and reasonable calculation basis is provided by the authors of [10]. Tao and others discussed the feasibility of introducing the balanced scorecard into the public sector for performance management based on the specific situation of government public management and the implementation environment of performance management, in order to gradually establish a scientific government performance appraisal system [11]. Nassar and Hosny used expert consultation and a survey to construct an integration of objective index evaluation, expert review, and public satisfaction measurement, including 5 first-level indicators and 14 second-level indicators such as system construction, process assurance, goal achievement, rule of law cost, and result satisfaction. This indicator system has a wide range of adaptability and verifiable scientific basis [12]. Edwards proposes an open and dynamic evaluation model based on fuzzy cluster analysis according to the purpose and requirements of project management performance evaluation and expounded its research ideas and framework [13]. Bamini studies the performance evaluation of public administration departments based on data mining technology. It uses the association rule data mining method of data mining technology to mine the performance-related data of the public administration department, and the association rule data mining method uses the three indicators of support, confidence, and association degree to mine the association rules between the data and establishes the performance evaluation system of the public administration department [14]. In order to save the cost of performance management and improve the efficiency of performance feedback and enterprise performance, Grossi et al. tried to introduce the ID3 algorithm in the decision tree method based on the hierarchical evaluation method [15]. Paul et al. applied entropy theory to public management and studied the disorder of public management, poor information, and poor operating conditions in the development process of public management, which led to internal friction, low efficiency, and excessive management costs in public management, high management goal drift or misalignment, friction and conflict in interpersonal relationships, and the decline of the entire public management system [16]. Kamaruddin and Abeysekera suggested a better data envelopment analysis algorithm. This algorithm fixes the data envelopment analysis inherent flaw of the algorithm of “relative effectiveness” in addition to avoiding the abnormal influence of weights. Theoretically, it is fairly complete to use this method to assess public sector performance, and the evaluation findings are well in line with the outcomes [17]. The financial performance of businesses was evaluated using the fuzzy clustering method by Brinkerhoff and Wetterberg, and the results are reasonable and supported by science [18].

In terms of practical application, the conventional public management performance evaluation method is flawed. This paper proposes and develops a fuzzy clustering-based performance evaluation model for public management based on research in the related literature. This paper ultimately develops an evaluation index system of first-level indicators and second-level indicators through the analysis of the organizational system, the technical system, the institutional mechanism, result orientation, and public satisfaction, as well as the research of related indicators. The fuzzy comprehensive evaluation method is used to realize public management performance evaluation by establishing the judgement matrix, computing weights, and building a fuzzy comprehensive evaluation model, in accordance with the established index system of public management performance evaluation. The analysis demonstrates that the research method can highly practically evaluate the performance of public administration departments.

## 3. Methodology

### 3.1. The Target Orientation and the Index System of Public Management Performance Evaluation

Where there is an organization, there is management and evaluation, and “promoting construction by evaluation” conforms to the incentive principle of management. The public management system is an open dissipative system, which is far from the equilibrium state and is characterized by stages. The public management system is also a multilevel, multifactor, open, and complex system [19], which is far from equilibrium, and there must be nonlinear effects among the various elements. The rule of law is the basic path for the transformation of government functions. Government performance evaluation of rule of law pursues the credibility of the government rule of law and pays attention to the realization of value goals. Specifically, it involves three important issues: (1) the relationship between government credibility and government executive power; (2) the relationship between democracy and rule of law; (3) measurement of the goal of the government ruled by law. An index is a kind of quantitative data, which is a set of the statistical data system. It is used to describe the index of social conditions, make social planning and social analysis [20], and make an evaluation of the present situation and the future. In fact, when evaluating the performance of public management by using the index system as an evaluation method, it is not always quantifiable, nor should it be quantified simply. Administration according to law and public management is influenced by various factors, and the performance index system of public management must be a scientific, rational, and logical organic whole. Perfect performance management should include five links: performance index system design, performance target system design, performance guidance and monitoring, performance evaluation, and performance feedback and improvement. Among them, the design of the performance index system is particularly important. Key performance indicators and the balanced scorecard are commonly used in this link. This paper holds that the performance evaluation of the government ruled by law forms a matrix structure with the performance evaluation of the government as a whole, government departments, government expenditures, and government policies. The organizational system, the technical system, the institutional mechanism, and other elements contained in the evaluation system are consistent with the performance evaluation of public management. Public management is a complex system process from concept to action, from local to global. The evaluation of public management is to better practice public management [21]. The public management performance orientation emphasizes the result orientation and the public satisfaction orientation. It is not limited to one-way evaluation from top to bottom but also pays more attention to public participation, reflecting the spirit of democracy and the rule of law and the essential relationship between the government and the public.

The indicators to be evaluated in the public management performance evaluation system cover a broad spectrum. The calculation of evaluation results is extremely difficult due to the completely different weights assigned to the evaluation indexes and evaluation requirements, and information sources used to gather the evaluation data, data calculation techniques, and quantitative indexes of the evaluation data. Both the evaluation subject and the index system, to a certain extent, determine the evaluation's credibility and scientific rigour, but they both support the evaluation's target orientation. Public management performance evaluation indicators can be categorised into subjective and objective indicators from the standpoint of the index system structure. They can also include qualitative, quantitative, characteristic, and supporting evaluation rules. We need to understand a number of relationships, such as those between quantifiable and nonquantifiable, subjective and objective evaluation, and reasonable and optimal evaluation, to transform the performance evaluation of the law-governed government from what it should be into what it is. The establishment of the index system serves as the foundation for assessing the state of public management, its contribution, the requirement for a dynamic evaluation of public management, and the requirement for the evaluation results to accurately reflect the situation. The degree of cooperation among the functions directly determines the efficiency of public management because public management is an organic whole made up of interrelated and interacting functions. The impact of performance-oriented target evaluation on the index system includes (1) requirement of indicators to reflect the dual functions of evaluation, evaluation of the current situation, encouragement of progress, and promotion of construction. (2) The index system should reflect the performance orientation and highlight the special status of key index evaluation, social response, and public satisfaction. (3) The index system should correspond to the target requirements of the outline of building a government under the rule of law and become the booster and vane for realizing the goal of a government under the rule of law. When establishing the evaluation index system, it should conform to the principles of consistency between the index and the evaluation target, compatibility with the index in the system, and relative independence of each evaluation index. At the same time, it should be designed according to the principles of measurability, completeness, and feasibility. In order to improve the resolution and representativeness of evaluation indexes, qualitative and quantitative analysis should be combined. The evaluation index system of public management performance is shown in Table 1.

The purpose of public management performance evaluation is to reflect the advantages of public resource investment as well as measure the government's work accomplishments using the concept of performance evaluation. The evaluation results will also show the government exactly where the issues are with the internal operations. The main concerns with evaluation are the target orientation and the index system. The mechanism for the evolution of public management systems includes both induction and fluctuation, with fluctuation acting as an inducer of evolution. Because of its openness, the public management system is affected by both internal and external fluctuations, meaning that it experiences both types of fluctuations. The public management system is evolving, but there is a mechanism for bifurcation. The index system is significantly influenced by the target orientation of public management performance evaluation; that is, various target orientations use various index systems. From an empirical perspective, the technical system is at the center of the evaluation system, but it is merely a tool used to farther the objectives of the evaluation. The cost-benefit economics model is the better approach to take when assessing the effectiveness of public management. It is thought to be a multiobjective decision-making problem with a variety of inputs and outputs. The data envelopment analysis algorithm's inherent, insurmountable limitation, however, is relative effectiveness. The so-called “relative effectiveness” refers to comparing the performance of the same departments when evaluating them and finally selecting the one with the best performance as the effective decision-making unit of DEA. Therefore, the performance of the evaluated department itself is not very good, but the DEA-effective results can still be evaluated according to the data envelopment analysis algorithm. This is inconsistent with the actual evaluation requirements. This paper puts forward a performance evaluation model of public management based on fuzzy cluster analysis and establishes an evaluation index system. This realizes the objective analysis and evaluation of the whole process of public management and provides a valuable basis for managers to carry out public management scientifically and reasonably.

### 3.2. Construction of the Public Management Performance Evaluation Model

The task of public performance analysis and evaluation is to analyze, process, and synthesize the collected data according to the purpose, standards, and methods of evaluation. The evaluation method is a commonly used analysis and evaluation method. This method has the advantages of simplicity and easy operation, but it has significant defects in performance feedback [22]. This chapter uses the fuzzy clustering method to analyze and evaluate the comanagement performance. The fuzzy clustering method is a method of classifying objective things by establishing fuzzy similarity relations. The characteristics of its classification [23] are the conclusion of fuzzy clustering does not indicate that objects absolutely belong to a certain class and do not belong to a certain class but indicates to what extent objects belong to a certain class and another class with a clear *λ* value. The composition and the algorithm flow of the fuzzy clustering system are shown in Figure 1.

Public management cost, internal management of public management, and learning and development of public management institutions are the input indices of public management, and public management performance is the output index of public management performance. After determining the weight of each index in the index system, it is necessary to establish a scoring standard for each evaluation index. This standard is determined using the fuzzy mathematics five-point scoring method, and a fuzzy comprehensive evaluation model is then built. By using fuzzy clustering, the content indicators are first grouped, and the properties and traits of each observer are known, as well as the causes of their similarities and differences. The classification results can then be compared to the current situation in order to identify any differences, which allow us to evaluate and comprehend the observer's growth and changes objectively. From there, we can make statistical inferences and predictions about the state of the series in the future, which can support project management decisions. According to the purpose and requirements of public management performance evaluation, we must first set the equation as follows:

(1) $$\begin{array}{c} X=\left\{x_{1},x_{2},x_{3},\ldots ,x_{n}\right\}. \end{array}$$

Each *x*_*i*_ has *u* evaluation indicators

(2) $$\begin{array}{c} x_{i}=\left\{x_{i1},x_{i2},x_{i3},\ldots ,x_{iu}\right\},\;i=1,2,3,\ldots ,u. \end{array}$$

The evaluation index system refers to the collection of various characteristics involved in the evaluation object. Data standardization is to standardize the data representing statistical indicators so as to facilitate analysis and comparison, as shown in the following equation:

(3) $$\begin{array}{c} x_{ij}^{\prime }=\frac{\left(x_{ij},{\bar{x}}_{i}\right)}{\delta_{i}},\;\left(i=1,2,3,\ldots ,n\;j=1,2,3,\ldots ,m\right). \end{array}$$

In the formula, *x*_*ij*_ is the original data, ${\bar{x}}_{i}$ is the average value of the original data, *δ*_*i*_ is the standard deviation of the original data, and *x*_*ij*_′ is the standardized data. The formula is expressed as follows:

(4) $$\begin{array}{c} {\bar{x}}_{i}=\frac{1}{n}\sum_{i=1}^{n}x_{ij},\delta_{i}=\frac{\sqrt{\sum_{i=1}^{n}{\left(x_{ij}-{\bar{x}}_{i}\right)}^{2}}}{n}. \end{array}$$

We standardize the data with the extreme value standardization formula and compress it to the [0,1] closed interval to achieve the same measurement effect, as shown in the following formula:

(5) $$\begin{array}{c} x_{ij}^{\prime \prime }=\frac{x_{ij}^{\prime }-x_{\min}^{\prime }}{x_{\max}^{\prime }-x_{\min}^{\prime }}. \end{array}$$

In the formula, *x*_max_′ is the largest in the original data set and *x*_min_′ is the smallest in the original data set.

(6) $$\begin{array}{c} \text{When }x_{ij}^{\prime }=x_{\max}^{\prime },\\ x_{ij}^{\prime \prime }=1,\\ \text{When }x_{ij}^{\prime }=x_{\min}^{\prime },\\ x_{ij}^{\prime \prime }=0. \end{array}$$

The formula for judging each column element in the normalized matrix is as follows:

(7) $$\begin{array}{c} F_{ij}=\frac{F_{ij}}{\sum_{k=1}^{m}F_{kj}},\;i,j=1,2,3,\ldots ,m. \end{array}$$

We add all the rows in the judgement matrix to obtain the normalization formula of each column of the judgement matrix as follows:

(8) $$\begin{array}{c} W_{i}=\sum_{j=1}^{m}F_{ij}. \end{array}$$

The *W*_*i*_=*W*_*i*_/∑_*j*=1_^*m*^*W*_*j*_ method is used to normalize each indicator vector, and the obtained result is the weight vector, which is as follows:

(9) $$\begin{array}{c} W=\left\{W_{1},W_{2},W_{3},\ldots ,W_{m}\right\}. \end{array}$$

The formula for calculating the average evaluation value is as follows:

(10) $$\begin{array}{c} B=W\circ R. \end{array}$$

When *B*_*j*_=1, the average evaluation value needs to be normalized by *B*_*i*_=*B*_*i*_/*B*_*j*_; the obtained result is

(11) $$\begin{array}{c} B=\left\{B_{1},B_{2},B_{3},\ldots ,B_{m}\right\}. \end{array}$$

The formula for calculating the final score value of the indicator *X*_*i*_ is as follows:

(12) $$\begin{array}{c} D=B\circ \left\{V_{1},V_{2},V_{3},\ldots ,V_{n}\right\}. \end{array}$$

We performed mathematical computations so as to realize the final evaluation of public management performance.

An index weight is an important content of the index system construction and should follow the principles of systematicness, typicality, independence, comparability, and operability. The weight of the index can be obtained by the AHP or structural equation model. The AHP is a decision-making method that decomposes the elements related to decision-making into objectives, criteria, schemes, and other levels and then makes qualitative and quantitative analysis on this basis. It mainly applies network system theory and the multiobjective comprehensive evaluation method. The AHP is characterized by its systematicness, conciseness, practicality, and less quantitative data. For example, using the structural equation model method, according to the path and factor load of variables in the empirical model of public management, the weight of each index can be obtained. From the perspective of index setting and weight allocation, the content of the second-level index only systematically sums up and summarizes the related work so as to guide the evaluation subject to evaluate the related work. Therefore, it is particularly important to design the third-level index in combination with the actual situation in different places, which needs to be completed in combination with practice. The standard coefficient is a horizontal parameter determined corresponding to the standard value of the fifth grade, which objectively reflects the different levels of the evaluation standard value, so as to accurately calculate the actual score of the performance evaluation quantitative index of the demonstration center.  Figure 2 shows the evaluation model architecture.

In this paper, the statistical threshold is combined with the actual needs and experience of project management, and the qualitative evaluation and quantitative measurement are combined so that the results can reflect the specific situation of the project management, and the monitoring and assessment data of different time points with the same nature are classified so as to facilitate the analysis and evaluation of project managers. Quantifying fuzzy data and comprehensively calculating mixed data are a key problem in the performance evaluation system. We find out the most discriminating attributes and divide the data into multiple subsets. Then, we find out the most discriminating attribute of each subset and then divide the data until all subsets only contain the same type of data. The evaluation results are weighted, and the concrete evaluation results are obtained by operation. With the dynamic change of indicators and the real-time update of data information, the applicability of the analysis model is improved through continuous simulation.

## 4. Result Analysis and Discussion

Public management performance evaluation is inherently quantitative, and the development of an index system depends on new developments in research methodology. The index system serves as both the technical means for achieving the evaluation goals and the central concern for those who evaluate public management. The public management department of a city is chosen as the experimental object in this section's attempt to determine the efficacy of the fuzzy clustering-based method for evaluating public management performance. From 2019 to 2021, this public administration department's relevant public management data totaled 3,015,427 pieces, which were gathered via the network. This section uses information technology to procedurally and functionally make the model, combining different clustering algorithms that can satisfy various evaluation requirements and comparing the potential differences among algorithms to realize the refinement and quantification of performance evaluation.  Figure 3 shows the learning performance curve of the algorithm.

From the analysis of the data shown in Figure 3, it can be concluded that the network in this paper can achieve the predetermined performance goal faster. It shows that the model constructed in this paper is effective. In order to strengthen the accuracy and reliability of the obtained results, this paper uses different data sets for simulation analysis. The results are shown in Table 2.

The results show that the highest accuracy of this clustering method can reach about 96%, and its accuracy is about 10% higher than the ID3 algorithm. The public performance evaluation model should strengthen the accumulation and collation of original data and establish a knowledge base according to the actual situation. At the same time, combining a series of methods such as factor analysis, correlation analysis, regression analysis, and principal component analysis continuously enriches and improves the evaluation system and methods, thereby improving the overall evaluation effect and efficiency. To test the evaluation performance of this method applied to the performance of public administration departments, the Kernighan–Lin algorithm and the *K*-means algorithm are selected as comparison methods, and the evaluation time of different methods in different data sizes is counted.  Figure 4 shows the running efficiency comparison of different algorithms.

From the experimental results shown in Figure 4, it can be seen that the efficiency of this method in evaluating the performance of public administration departments is higher than that of the other two algorithms. The real-time evaluation of this method is obviously higher than that of the other two methods, and it can be applied to the performance evaluation of public administration departments with a large amount of data. Meanwhile, the algorithm has high practicability. Comparing the accuracy of different algorithms, the results are shown in Figure 5.

The fuzzy comprehensive evaluation method is used to evaluate the performance of public management based on the mining results, and the experimental accuracy results show that this method can effectively evaluate the performance of public management. This method is scientific, reasonable, and practical and can achieve fairness and justice in evaluation and has high applicability. The error comparison of different algorithms is shown in Figure 6.

The experimental results show that the algorithm error is small. This method can effectively obtain the results of public management performance evaluation. The evaluation results can be applied not only to the performance comparison of public administration departments in different provinces and cities but also to the performance comparison of employees in public administration departments. According to the evaluation results, public administration departments can judge the reasons that affect the performance evaluation results of public administration departments and formulate corresponding improvement measures to improve the management level of public administration departments. The comparison between the predicted value and the actual evaluation value is shown in Figure 7.

The public management performance evaluation model is a dynamic and changing structure, and there are also differences and uncertainties in the specific implementation of management. It is undoubtedly a very important aspect how to establish a complete, systematic, and feasible performance evaluation standard under the government's set objectives. The experimental results of this section show that the fuzzy clustering method can effectively analyze and evaluate the comanagement performance, and this method is scientific and practical.

## 5. Conclusions

The key to advancing the rule of law is to establish a government that is governed by the law. This is also a crucial step in making the rule of law a reality. The construction of government must always be performed with the rule of law in mind. Law-abiding administration must be vigorously promoted, and the government work's level of legalisation, standardization, and proceduralization must always be raised. Establishing and implementing public performance management is crucial to creating a modern, democratic, effective, fair, and honest government. It also involves changing the management style of the system that is used to evaluate the performance of the government and its public servants. This study examines the shortcomings of the current public management performance evaluation system, proposes a fuzzy clustering-based public management performance evaluation model, and explains the guiding principles of this approach. This paper ultimately develops an evaluation index system of first-level indicators and second-level indicators through the analysis of the organizational system, the technical system, the institutional mechanism, result orientation, and public satisfaction, as well as the research of related indicators. The fuzzy comprehensive evaluation method is used to realize public management performance evaluation by establishing the judgement matrix, computing weights, and building the fuzzy comprehensive evaluation model, in accordance with the established index system of public management performance evaluation. According to the research, this clustering method can achieve an accuracy as high as 96 percent, which is about 10% higher than the accuracy of the ID3 algorithm. This demonstrates how well this method can assess the efficiency of public administration divisions and how highly practicable it is. In the next step, this paper will focus on enhancing the correlation and the membership degree of indicators. By combining subjective and objective evaluation, the index system is fully optimized to reduce the system error. We optimize and improve the index system through further practice tests.

## Figures and Tables

**Figure 1:** Composition and algorithm flow of the fuzzy clustering system.

**Figure 2:** Evaluation model architecture.

**Figure 3:** Learning performance curve of the algorithm.

**Figure 4:** Comparison of results of running efficiency of different algorithms.

**Figure 5:** Comparison of accuracy of different algorithms.

**Figure 6:** Error comparison of algorithms.

**Figure 7:** Comparison between the predicted value and the actual evaluation value.

**Table 1:** Public management performance evaluation index system.

Index system	First-class evaluation index	Secondary evaluation index
Public management performance evaluation index system	Ability level	Expression level
		Professional skill
		Investigation level
		Innovation level
		Independent working level
		Communication level
	Moral level	Political level
		Conscientiousness
		Sense of competition
		Affinity
		Professional ethics
		Self-discipline level
	Functional mode	Workload
		Attendance rate
		Work efficiency
		Working degree
		Information publicity
	Public satisfaction	Administrative service
		Administrative supervision
		Service and image
		Prevention and resolution of social contradictions

**Table 2:** Clustering accuracy results of different algorithms on different data sets.

Algorithms	Precision		
	Data set A	Data set B	Data set C
Kernighan–Lin algorithm	0.841	0.863	0.871
*K*-means algorithm	0.783	0.841	0.798
*K*2 mean algorithm	0.735	0.796	0.764
ID3 algorithm	0.861	0.864	0.866
Fuzzy clustering algorithm	0.963	0.967	0.961

## Data Availability

The data used to support the findings of this study are available from the corresponding author upon request.
